The article "Upregulation of CCT-3 Induces Breast Cancer Cell Proliferation Through miR-223 Competition and Wnt/β-Catenin Signaling Pathway Activation" was retracted in 2025. Reasons: original data or images not available; unreliable results or conclusions; concerns about the data; concerns about the images.

# Upregulation of CCT-3 Induces Breast Cancer Cell Proliferation Through miR-223 Competition and Wnt/β-Catenin Signaling Pathway Activation

**DOI:** 10.3389/fonc.2020.533176

**Published:** 2020-09-24

**Authors:** Hongbo Qu, Fang Zhu, Huaying Dong, Xiongqiang Hu, Mingli Han

**Affiliations:** ^1^Department of Breast and Thyroid Surgery, The First People's Hospital of Chenzhou, Chenzhou, China; ^2^Department of Breast Health Center, The First People's Hospital of Chenzhou (South Hospital), Chenzhou, China; ^3^Department of General Surgery, Hainan General Hospital, Hainan Medical University, Haikou, China; ^4^Department of Breast Surgery, The First Affiliated Hospital of Zhengzhou University, Zhengzhou, China

**Keywords:** ceRNA, miR-223, Wnt/β-catenin, breast cancer, CCT-3

## Abstract

The clinical significance and the function of chaperonin-containing TCP1 complex 3 (CCT-3) in breast cancer remain unknown. In this study, we found that CCT-3 was markedly overexpressed in breast cancer tissues. Statistical analysis revealed a significant correlation of CCT-3 expression with advanced breast cancer clinical stage and poorer survival. Ablation of CCT-3 knocked down the proliferation and the tumorigenicity of breast cancer cells *in vitro* and *in vivo*. CCT-3 may regulate breast cancer cell proliferation through a ceRNA network between miR-223 and β-catenin, thus affecting Wnt/β-catenin signaling pathway activation. We also validated that CCT-3 and β-catenin are novel direct targets of tumor suppressor miR-223. Our results suggest that both mRNA and the protein levels of CCT-3 are potential diagnosis biomarkers and therapeutic targets for breast cancer.

## Introduction

Breast cancer is the most frequently diagnosed cancer and the leading cause of cancer death among females, accounting for 23% of total cancer cases and 14% of cancer deaths (based on the GLOBOCAN 2008 estimates, about 12.7 million cancer cases and 7.6 million cancer deaths are estimated to have occurred in 2008) (1). Protein-coding gene expression profiling, such as estrogen receptor (ER)+, Triple negative, and human epidermal growth factor receptor (HER)2+, helps in addressing breast cancer clinical treatment (2). A diagnosis in the early stages enables better and higher cure rate and longer survival rate. However, the identification of early breast cancer events is far from being achieved. Thus, identifying a potential early biomarker is of high clinical value.

The chaperonin-containing TCP1 complex (CCT) is also called the TCP1 ring complex (TRiC), from a 1-MDa hetero-oligomeric complex that mediates ~10% of newly synthesized protein. The CCT proteins are folded in an ATP-dependent manner (3). The CCT family complex consists of two ring regions; each region is composed of radially arranged subunits including CCT1–CCT8. The CCT family members have been shown to be involved in tumorigenesis recently. Overexpression of CCT-2, CCT-5, and CCT-6 has been reported in colorectal cancer and was linked to poor prognosis (4, 5). In hepatocellular carcinoma, CCT-3, and CCT-8 have been proven as oncogenes that promote cancer cell proliferation (6, 7). Notably, CCT-1 and CCT-2 are essential for the survival of breast cancer cells that make them susceptive oncogenes (8–11). However, the clinical relevance and the function of CCT-3 in breast cancer remain largely unclear.

The article "Upregulation of CCT-3 Induces Breast Cancer Cell Proliferation Through miR-223 Competition and Wnt/β-Catenin Signaling Pathway Activation" was retracted in 2025. Reasons: original data or images not available; unreliable results or conclusions; concerns about the data; concerns about the images.

We aim to unveil the clinical significance of CCT-3 and its role in breast cancer in this study. We found that CCT-3 overexpressed significantly in breast cancer tissues. The upregulation of CCT-3 was associated with poor clinical prognosis of breast cancer. Further mechanistic investigations into the function of CCT-3 in breast cancer were performed through gain- and loss-of-function studies, through which we found that CCT-3 can promote breast cancer cell proliferation and tumorigenicity via β-catenin nuclear accumulation and miR-223 inhibition. Our results offer a potential diagnosis biomarker and therapeutic target for breast cancer.

## Materials and Methods

### Reagents

Anti-CCT3, anti-β-catenin, anti-cyclinD1, anti-c-Myc, anti-lamin B, and anti-GAPDH were from Abcam (Cambridge, UK). Anti-GSK3β and anti-phospho-GSK3β were purchased from Cell Signaling Technology (Danvers, USA). The dual-luciferase reporter assay system, including PGL3-Basic and PRL-TK vectors, was from Promega Corporation (Wisconsin, USA). miRNA mimics and siRNAs were purchased from Biomics Biotechnologies (Nantong, China).

### Cell Lines

The cell lines MDA-MB-231, MDA-MB-468, MCF-7, and ZR-75-1 were purchased from Cell Bank of Type Culture Collection of Chinese Academy of Sciences (Shanghai, China) and cultured in 10% fetal bovine serum Dulbecco's Modified Eagle's Medium (Thermo Fisher Scientific, USA).

### Plasmid, Lentivirus, and Cell Transfections

A CCT-3 expression construct was generated by cloning synthesized full-length human CCT-3 cDNA into Ubi-MCS-3FLAG-SV40-puromycin lentiviral vectors (Genechem Company, Ltd., Shanghai, China). The overexpression vector does not contain the UTRs of CCT-3. The hU6-MCS-CMV-puromycin lentiviral vectors were also from Genechem Company, Ltd., and were used to knock down the CCT-3 expression. The target sequences are siRNA-1: GCCAAGTCCATGATCGAAATT and siRNA-2: GAGATGAATACTTTACTTTCATC. The negative control lentiviral vector was used without a shRNA sequence.

A CCT-3 3′UTR expression vector was produced by cloning synthesized full-length human CCT-3 3′UTR into PCDNA 3.1(+).

The article "Upregulation of CCT-3 Induces Breast Cancer Cell Proliferation Through miR-223 Competition and Wnt/β-Catenin Signaling Pathway Activation" was retracted in 2025. Reasons: original data or images not available; unreliable results or conclusions; concerns about the data; concerns about the images.

The dual-luciferase reporter was constructed by synthesizing a full-length wild-type CCT-3 3′UTR (containing miR-223 binding site), and a mutant CCT-3 sequence (mutant in miR-223 binding site) was cloned into PGL3-Basic vector. These vectors were appointed, respectively, as PGL3-Basic-wt-CCT-3 and PGL3-Basic-mut-CCT-3.

The miRNA mimics, inhibitors, and plasmids were transfected by using Lipofectamine 2000 (Invitrogen, California, USA).

For the generation of the knockdown CCT-3 cell lines, the lentivirus contains CCT-3 siRNA sequence, and control sequences were added to the breast cancer cells, respectively. After 48 h of infection, the cells were analyzed by Western blot (WB) to detect the CCT-3 protein level. For CCT-3-overexpressed cell lines, lentivirus containing CCT-3 full-length cDNA sequence was added to the breast cancer cells, and the overexpression effect was verified by Western blot.

### Patient Samples

Two independent cohorts were used in this study:

Cohort 1: 258 formalin-fixed and paraffin-embedded (FFPE) breast cancer samples were histopathologically and clinically diagnosed at The First People's Hospital of Chenzhou from 2005 to 2019.

Cohort 2: 43 pairs of fresh breast cancer and adjacent non-cancerous tissues were collected from patients who were diagnosed with breast cancer between 2017 and 2019 at The First People's Hospital of Chenzhou.

The TNM classification depends on the American Joint Committee on Cancer staging system (12). The ER, progesterone receptor (PR), and HER2 classification was according to the American Society of Clinical Oncology/College of American Pathologists Guideline Recommendations (13, 14).

Samples were scored using the immunohistochemical score (his) value as described by Soslow (15): IHS = A × B, where A is the percentage of positive cells and B is the positive cell staining intensity grade. B was scored from 0 to 3 as follows: 0, negative; 1, low positive; 2, medium; and 3, strong positive. Score ≤1 indicates low expression. Score >1 indicates high expression.

Patient information is presented in Supplementary Table 1.

### Animals

Nude mice (about 4–6 weeks) were raised under specific-pathogen-free conditions. For subcutaneous implantation, 5 × 10^6^ lenti-siRNA and lenti-negative control (NC)-treated cells suspended in 100 ul PBS were injected subcutaneously into BALB/C nude mice. The tumors were examined every 4 days. On day 28, the mice were euthanized, and tumor volume and tumor weight were measured.

### Western Blotting

The cellular proteins of CCT-3 knockdown and overexpressing cells and control cells were extracted and separated in sodium dodecyl sulfate- polyacrylamide gel electrophoresis gels. CCT-3 knockdown and overexpressing cell and control cell proteins were IB analyzed. The host gene GAPDH on the same sample was used as a loading control.

The article "Upregulation of CCT-3 Induces Breast Cancer Cell Proliferation Through miR-223 Competition and Wnt/β-Catenin Signaling Pathway Activation" was retracted in 2025. Reasons: original data or images not available; unreliable results or conclusions; concerns about the data; concerns about the images.

### RNA Extraction and Quantification

Total RNA was extracted with Trizol (Invitrogen, California, USA). The primers used for real-time PCR for CCT-3 are as follows: CCT3-F: CCTCCAGGTATCTTTTCCACTCT; CCT3-R: TCAGTCGGTGGTCATCTTTGG; GAPDH-F: TGACTTCAACAGCGACACCCA; GAPDH-R: CACCCTGTTGCTGTAGCCAAA. Has-miR-223-3p expression was quantified by using miDETECT A Track hsa-miR-223-3p Forward Primer kit (Ruibo, Guangzhou, China). The protocols of reverse transcription and quantification were followed as per the manual.

### MTT Assay

CCT-3 knockdown and overexpressing cells and control cells were seeded at a density of 1 × 10^3^ cells per well in 96-well plates. The viability of CCT-3 knockdown and overexpressing cells and control cells was assessed by MTT assay for 5 days.

### Colony Formation Assay

CCT-3 knockdown and overexpressing cells and control cells were seeded at a density of around 200–400 cells in one 6-cm cell culture dish. The CCT-3 knockdown and overexpressing cells and control cells were cultured for 2 weeks. Colonies from CCT-3 knockdown and overexpressing cells and control cells were stained with crystal violet (1%), photographed, and counted.

### Flow Cytometry

The CCT-3 knockdown and overexpressing cells and control cells were fixed with 70% ethanol overnight at 4°C. They were then stained with propidium iodide and analyzed with a FACScan flow cytometer (BD, Biosciences, San Jose, CA, USA). The data were analyzed by ModFit 3.0 software (Verity Software House, Topsham, USA).

### Immunofluorescence

The CCT-3 knockdown and overexpressing cells and control cells were fixed (4% paraformaldehyde), permeabilized (0.25% Triton), and incubated at 4°C overnight. Then, they were incubated with rhodamine-conjugated goat antibodies against rabbit IgG (Abcam, Cambridge, UK). Nuclei were stained with DAPI.

### Top Flash Reporter Assay

Wild-type and mutant TOP/FOP flash β-catenin LUC reporter (Addgene, Inc., Cambridge, MA, USA) was co-transfected with siRNA and miRNA. The transfection was performed according to the manufacturer's protocol. A luciferase activity assay was carried out 48 h after transfection and assayed for relative luciferase activity normalized with Renilla values.

### Statistical Analysis

Overall survival curves were calculated using Kaplan–Meier and log-rank tests. Mann–Whitney test (*U*-test) was used in CCT-3 mRNA and miR-223 expression and clinicopathological characteristics. Student's *t*-test was used in analyzing further experiment results such as those of MTT assay, dual-luciferase activity, and so on. *p* < 0.05 was considered to be statistically significant.

The article "Upregulation of CCT-3 Induces Breast Cancer Cell Proliferation Through miR-223 Competition and Wnt/β-Catenin Signaling Pathway Activation" was retracted in 2025. Reasons: original data or images not available; unreliable results or conclusions; concerns about the data; concerns about the images.

## Results

### CCT-3 Is Significantly Upregulated in Breast Cancer Tissues

The WB results indicated that CCT-3 has a strong expression of both mRNA and protein levels in five breast cancer cell lines: MDA-MB-231, MDA-MB-468, MCF-7, ZR-75-1, and T47D (Figures 1A,B). In addition, the expression of CCT-3 protein in tumor tissue was significantly higher than that in normal tissue (Figure 1A). Furthermore, the protein expression levels of CCT-3 in FFPE breast cancer tissues and their corresponding non-tumorous tissues showed that CCT-3 is also overexpressed in breast cancer tissues (Figure 1C). These findings indicate that CCT-3 is upregulated in breast cancer.

**Figure 1:** CCT-3 is upregulated in breast cancer. **(A)** Protein levels of CCT-3 in five breast cancer cell lines (left) and in matched primary breast cancer tissues (T) and corresponding non-tumorous tissues (NT; right). **(B)** RNA levels of CCT-3 in five breast cancer cell lines. **(C)** Immunohistochemistry (IHC) staining analysis of CCT-3 protein expression in matched primary breast cancer tissues (T) and corresponding non-tumorous tissues (NT). **(D)** Kaplan–Meier curves with univariate analyses (log-rank) for patients with breast cancer with low CCT-3-expressing (*n* = 152) vs. high CCT-3-expressing tumors (*n* = 106). **(E)** IHC staining analysis of CCT-3 protein expression in breast cancer tissues from clinical stages I to IV. **(F)** Mann–Whitney test for CCT-3 expression in 43 pairs of breast cancer tissues (T) and their corresponding non-tumorous tissues (NT) (frozen samples).

### CCT-3 Expression Is Correlated With Breast Cancer Progression

To further establish the clinical importance of CCT-3 in breast cancer, we analyzed 258 breast cancer FFPE tissues by immunohistochemistry staining. The relationship between CCT-3 protein expression and breast cancer clinical features, including age, clinical stage, TNM classification, expression of estrogen receptor, expression of progesterone receptor, and expression of HER2, was analyzed.

As shown in Figure 1D, the K–M survival curves and the log-rank test survival analysis revealed that the overall survival of patients with high levels of CCT-3 was significantly poorer than those who with low CCT-3 levels (Figure 1D, *p* < 0.001).

Furthermore, CCT-3 expression in breast cancer increased with advanced clinical stage (Figure 1E). The poor pathologic differentiation was also related with a high expression of CCT-3. Moreover, Fisher's exact test analysis revealed that the CCT-3 levels were significantly (*p* < 0.001) correlated with clinical stage, TNM classification, and PR expression (Supplementary Table 2).

The article "Upregulation of CCT-3 Induces Breast Cancer Cell Proliferation Through miR-223 Competition and Wnt/β-Catenin Signaling Pathway Activation" was retracted in 2025. Reasons: original data or images not available; unreliable results or conclusions; concerns about the data; concerns about the images.

Interestingly, we found that the mRNA expression levels were also upregulated in 43 fresh breast cancer tissues (Figure 1F, *p* < 0.001). Analogous results were obtained by analyzing the CCT-3 mRNA expression levels in The Cancer Genome Atlas Cancer Genome (TCGA) breast cancer samples. As shown in Supplementary Figure 1A, the CCT-3 mRNA levels were also strongly overexpressed in 1,106 breast cancer tissues (*p* < 0.001) (16, 17). Strikingly, the results of K–M survival curves and log-rank test survival analysis in 3,553 breast cancer patients also showed a significant poor overall survival of high-CCT-3-mRNA-level patients (18).

Our result combined with TCGA data showed that both the mRNA and the protein levels of CCT-3 are upregulated in breast cancer and are correlated with poor overall survival. CCT-3 may be a diagnostic and prognostic biomarker for breast cancer.

### CCT-3 Promotes Breast Cancer Cell Tumorigenicity by Cell Cycle Regulation

The clinical significance of CCT-3 indicated that its overexpression may contribute to the proliferation of breast cancer cells. We next performed gain- and loss-of-function studies in two breast cancer cell lines to investigate the biological significance of CCT-3 expression in the regulation of breast cancer proliferation and development.

As shown in Figures 2A,B, the CCT-3 protein levels were elevated and reduced after expressing vector (OE) or interfering vectors (siRNA-1 and siRNA-2) infection in two cells. After 5 days, the MTT assay revealed that, compared with control cells (MDA-MB-231 OE-NC and T47D OE-NC), the proliferation rate was notably increased in CCT-3 overexpressed breast cancer cells (MDA-MB-231 OE and T47D OE). In contrast, significantly reduced cell viability was found in CCT-3 knockdown cells (MDA-MB-231 siRNA-1, MDA-MB-231 siRNA-2, and T47D siRNA-1 and T47D siRNA-2) (Figure 2C). The colony formation assays (Figure 2D) confirmed the results of the MTT assays.

**Figure 2:** CCT-3 promotes breast cancer cell proliferation and tumorigenicity *in vitro* and *in vivo*. **(A)** Protein levels of CCT-3 expression in CCT-3-overexpressed and CCT-3-silenced cells. MTT assays **(B,C)**, colony formation assay **(D)**, and flow cytometric analysis **(E)** indicated that the growth rates increased in CCT-3-overexpressed cells and decreased in CCT-3-silenced cells. The cells were arrested in G2/M phase when CCT-3-silenced. Values are mean ± SD of three independent experiments. ^##^*p* < 0.01 (OE vs. OE-NC), ***p < 0.001 (siRNA vs. siRNA-NC), *t*-test. **(F)** Tumors derived from the vector-infected and the CCT-3-silenced cells. Representative images of tumor growth (left). Tumor volume growth curves (middle). Mean tumor weight (right) at 28 days after inoculation. *p < 0.05, *t*-test.

The article "Upregulation of CCT-3 Induces Breast Cancer Cell Proliferation Through miR-223 Competition and Wnt/β-Catenin Signaling Pathway Activation" was retracted in 2025. Reasons: original data or images not available; unreliable results or conclusions; concerns about the data; concerns about the images.

Since cell proliferation can be regulated by CCT-3, we then hypothesized that cell cycle distribution may be different following CCT-3 overexpression or silencing (OE or siRNA-1 and siRNA-2). As shown in Figure 2E, G1/S arrest was observed in CCT-3-silenced cells (OE-NC and siRNA-NC). Meanwhile, CCT-3 overexpression resulted in the promotion of G1/S transition in MDA-MB-231 and T47D cells.

We then asked whether CCT-3 was in a position to promote breast cancer cell tumorigenicity *in vivo*. In nude mice, the control cells grew much faster than CCT-3-silenced breast cancer cells (siRNA-1 and siRNA-2). Moreover, tumors formed from CCT-3-silenced cells had less tumor weight and volume than siRNA-NC control tumors (Figure 2F).

These results demonstrated that CCT-3 deregulation may be a reason for breast cancer cell's uncontrolled proliferation *in vitro* and *in vivo*. Such effect may be carried out in a G1/S cell-cycle-regulative manner.

### Wnt/β-Catenin Is a Key Signaling Pathway Mediating CCT-3 Regulation

Wnt/β-catenin is a key signaling pathway in cancer cell proliferation, migration, and adhesion (19, 20). We tried to find correlations between CCT-3 expression and Wnt/β-catenin activity. Firstly, we employed TOP/FOP flash to evaluate the signal activity. Wnt signaling was highly activated in MDA-MB-231 and T47D cells when CCT-3 was upregulated, as shown in Figure 3A. In contrast, knocking down of CCT-3 knocked down the Wnt signaling significantly, which suggested that Wnt/β-catenin is a key signaling pathway mediating CCT-3 regulation in breast cancer cell proliferation.

**Figure 3:** CCT-3 promotes breast cancer cell proliferation through Wnt/β-catenin signaling pathway activation. **(A)** TOP/FOP flash indicated that the Wnt/β-catenin signaling pathway activation was regulated by CCT-3. Values are mean ± SD of three independent experiments. *p < 0.05, **p < 0.01 (OE vs. OE-NC), ^###^*p* < 0.001 (siRNA vs. siRNA-NC), *t*-test. **(B)** Protein levels of CCT-3, p-GSK-3β, GSK-3β, β-catenin (nucleus), cyclin D1, and c-Myc in CCT-3-overexpressed and CCT-3-silenced cells. Lamin B and GAPDH were used as loading controls. **(C)** The translocation of β-catenin from the cytoplasm to the nucleus was detected by immunofluorescence staining following CCT-3 overexpression and inhibition in breast cancer cells.

Importantly, we found that the protein level of p-GSK-3β and β-catenin nuclear accumulation increased in CCT-3-overexpressed MDA-MB-231 and T47D cells. CCT-3 also affected the expression levels of β-catenin downstream effectors such as cyclin D1 and c-myc (Figure 3B). Inversely, the signal transduction was knocked down in CCT-3-siRNA-treated breast cancer cells. The protein levels of cyclinD1 in CCT-3-overexpressed and CCT-3-silenced cells at least in part explained the G1/S modulation effect observed by fluorescence-activated cell sorting.

The article "Upregulation of CCT-3 Induces Breast Cancer Cell Proliferation Through miR-223 Competition and Wnt/β-Catenin Signaling Pathway Activation" was retracted in 2025. Reasons: original data or images not available; unreliable results or conclusions; concerns about the data; concerns about the images.

To further testify the nuclear accumulation of β-catenin, immunofluorescence was performed. As shown in Figure 3C, the nucleus β-catenin increased significantly when CCT-3 was upregulated.

These data implied that CCT-3 may promote breast cancer tumorigenesis at least in part via activating the Wnt/β-catenin signaling pathway.

### CCT-3 Regulates β-Catenin Expression Through miR-223 Competition

Coding protein transcripts exert biological function not only through canonical coding protein pathway but also through non-coding RNAs. miRNAs play important roles in regulating cancer proliferation, invasion, and migration. Coding protein can exert biological function through competing for functional miRNAs in 3′UTR (21). There are three miRNA binding sites in CCT-3 3′UTR, miR-24-3p, miR-128-3p, and miR-223, according to Targetscan 7.2 (http://www.targetscan.org/cgi-bin/targetscan/vert_72/view_gene.cgi?rs=ENST00000295688.3&taxid=9606&showcnc=0&shownc=0&shownc_nc=&showncf1=&showncf2=&subset=1). We found, in 43 pairs of breast cancer tissues, that miR-223 expression was significantly decreased in cancer tissues compared with corresponding non-tumorous tissues in 43 pairs of fresh samples (Figure 4A, *p* < 0.001). Moreover, in 770 TCGA breast cancer samples, the miR-223 expression levels were also notably lower in cancer tissues (Supplementary Figure 1C, *p* < 0.001).

**Figure 4:** CCT-3 promotes breast cancer cell proliferation through miR-223 suppression. **(A)** Mann–Whitney test for miR-223 expression in 43 pairs of breast cancer tissues (tumor) and their corresponding non-tumorous tissues (NT) (frozen samples). **(B)** Wilcoxon signed rank test for miR-223 and CCT-3 in 43 pairs of breast cancer tissues (tumor) and their corresponding non-tumorous tissues (NT) (frozen samples). **(C)** RNA levels of miR-223 in CCT-3-silenced, CCT-3-overexpressed, and CCT-3 3′UTR overexpressed cells. ***p < 0.001 (siRNA vs. siRNA-NC), ^##^*p* < 0.01 (CCT-3 3′UTR vs. OE-NC), *t*-test. **(D)** MiR-223 mimics and inhibitor significantly suppressed and upregulated the luciferase activity of wild-type CCT-3 3′UTR, respectively, *p < 0.05, ***p < 0.001, *t*-test. **(E)** Protein levels of CCT-3 in miR-223 mimics and inhibitor-treated cell. GAPDH was used as loading control. **(F)** MiR-223 mimics and inhibitor significantly suppressed and upregulated the luciferase activity of wild-type β-catenin 3′UTR, respectively; **p < 0.01, ***p < 0.001, *t*-test. **(G)** Protein levels of β-catenin in miR-223 mimics and inhibitor-treated cell. GAPDH was used as loading control. MTT assays indicated that miR-223 rescued the anti-proliferation effect of CCT-3 in MDA-MB-231 **(H)** and T47D **(I)**. **(J,K)** TOP/FOP flash indicated that the Wnt/β-catenin signaling pathway activation was regulated by miR-223 and CCT-3 3′UTR. Values are mean ± SD of three independent experiments. ***p < 0.001 (miR-223 vs. miR-NC), ^##^*p* < 0.01, ^###^*p* < 0.001 (miR-223 + CCT-3 3′UTR vs. miR-223), *t*-test.

The article "Upregulation of CCT-3 Induces Breast Cancer Cell Proliferation Through miR-223 Competition and Wnt/β-Catenin Signaling Pathway Activation" was retracted in 2025. Reasons: original data or images not available; unreliable results or conclusions; concerns about the data; concerns about the images.

Interestingly, we found a negative correlation of CCT-3 and miR-223 mRNA expression levels in 43 fresh breast tissues and 748 TCGA tissues (Figure 4B and Supplementary Figure 1D, *p* < 0.001).

To further investigate whether CCT-3 can modulate miR-223 expression, the CCT-3 3′UTR was therefore cloned into the multicloning site of a cytomegalovirus-driven expression plasmid. As predicted, the overexpression of 3′UTR, but not the coding region of CCT-3, markedly decreased miR-223 expression levels in both MDA-MB-231 and T47D cells. Similarly, silencing of CCT-3 increased the miR-223 expression levels dramatically (Figure 4C).

We then hypothesized that miR-223 can directly bind to the 3′UTR of CCT-3. A luciferase reporter in which the full length CCT-3 3′UTR was inserted into the PGL3-promoter vector was constructed. A mutant reporter was also constructed, in which the miR-223 seed region sequence in the complementary sites was changed. Our results showed the luciferase activity in the wild-type group. Moreover, luciferase activity was considerably decreased and increased in miR-223 mimics and inhibitor-treated group, respectively (Figure 4D, *p* < 0.01 and *p* < 0.05), suggesting that the CCT-3 is a direct binding target of miR-223. The modulating effect between miR-223 and CCT-3 was confirmed by Western blotting assays. Figure 4E shows that miR-223 mimics inhibited the CCT-3 protein expression, while blocking miR-223 with inhibitors elevated the CCT-3 protein level.

Notably, the anti-proliferation effect of miR-223 in two breast cancer cell lines was rescued by the overexpression of CCT-3 3′UTR (Figures 4H,I), which also supported the notion that CCT-3 regulates breast cancer cell proliferation through miR-223. There is also a miR-223 binding site predicted in the 3′UTR of β-catenin. Luciferase activity assay and Western blot assay indicated that β-catenin is a direct target of miR-223 (Figures 4F, G). The results of the TOP/FOP flash assay also showed a rescue effect of CCT-3 3′UTR on miR-223-induced Wnt signaling activation (Figures 4J,K).

The article "Upregulation of CCT-3 Induces Breast Cancer Cell Proliferation Through miR-223 Competition and Wnt/β-Catenin Signaling Pathway Activation" was retracted in 2025. Reasons: original data or images not available; unreliable results or conclusions; concerns about the data; concerns about the images.

Interestingly, we found that miR-223 upregulation was also able to inhibit Wnt/β-catenin activity, which can also be compensated by CCT-3 3′UTR overexpression.

Collectively, our results indicated that CCT-3 may promote breast cancer cell by directly binding to miR-223, thus weakening the regulation of miR-223 in the Wnt/β-catenin pathway.

## Discussion

Taken together, the findings of this study showed that both mRNA and CCT-3 protein and mRNA levels are substantially correlated with the clinical malignancy and prognosis of breast cancer. CCT-3 regulates breast cancer tumorigenesis by promoting cell proliferation and cell cycle progression. CCT-3 promotes cell proliferation by binding directly to miR-223, thus promoting β-catenin nuclear accumulation. To our knowledge, this study provides a new insight that both protein and mRNA of CCT-3 may play a vital role in breast cancer cell tumorigenesis and progression for the first time.

In order to form a tumor, cells must pass through a multistep process including uncontrolled signaling transduction, energy metabolism, cell growth, and tumor formation (22). These steps are essential, and each step has several barriers, which must be overcome by malignant cells for successful tumor formation. The malignant cells accumulate several manners of changes, including changes in protein coding and non-coding gene expression profiles, to overcome these barriers. Therefore, identification of abnormally expressed genes that lead to tumorigenesis is important for providing new diagnostic biomarkers and potential therapeutic targets.

CCT-3 was significantly upregulated in a large proportion of human breast cancer tissues, and its overexpression was also significantly correlated with breast cancer clinical characteristics, including the clinical stage and the TNM classification. Importantly, patients with low CCT-3 expression have better overall survival of 5 years, indicating that both CCT-3 mRNA and protein level are potential biomarkers for breast cancer patient prognosis.

CCT-3 has been reported to promote HepG2 cell proliferation (6). Stat3 and CCT-3 have been reported to modulate mutually by binding with each other. CCT-3 binds to the β-strand-rich, DNA binding domain of Stat3. CCT-3 modulated Stat3 expression levels and function by manipulating its interaction with Stat3 (23). Neef et al. reported that protein misfolding induced stress, and apoptosis-modulating gene heat shock transcription factor 1 is directly regulated by CCT-3 (24). The Wnt signal is a canonical pathway for cell fate determination. It is also a non-canonical pathway for cell migration, invasion, and polarity. Nuclear complex, including T-cell factors, β-catenin, PYGO, etc., activates WNT target gene transcription (25–27). The Wnt pathway component mutations and deregulation can induce a disease, especially cancer (28). However, no evidence had shown a relationship between CCT-3 and the Wnt/β-catenin pathway. In this study, we found that CCT-3 promotes β-catenin nuclear translocation. As a result, Wnt/β-catenin signaling was activated when CCT-3 was knocked down; the target genes downstream, such as cyclin D1 and c-myc, were then transcribed with the help of β-catenin. These Wnt/β-catenin target genes promote breast cancer cell G1/S transition and other oncogene transcriptions, keeping the malignant proliferative ability. The TriC/CCT complex tends to bind to a β-strand structure (29). The C-terminal of β-catenin is rich in β-strands (30). The immunofluorescence data in Figure 3C shows the co-localization of CCT-3 and β-catenin in breast cancer nucleus. Hence, there is a high possibility that CCT-3 may recruit β-catenin into the nucleus through direct binding. Co-immunoprecipitation between CCT-3 and β-catenin can be used to prove the precise mechanism.

miRNA response elements in coding and non-coding genes could compete with the miRNA target gene and regulate its expression. Such gene is called competing endogenous RNA (ceRNA), and the “RNA–miRNA” interaction appreciably extends the gene function product from protein to mRNA. Generally, non-coding RNAs such as LncRNA 2810403, CA7-4, and LncIRS1 are prone to exert biological function through ceRNA mechanism (31, 32). Recently, coding genes have also been proven to regulate cell proliferation through ceRNA network. CXCR4 3′UTR, a validated ceRNA in breast cancer, has been reported to promote cancer cell metastasis, proliferation, and survival by regulating miR-146a activity (33). Evidences show that miR-223 is a tumor suppressor gene in breast cancer. One of the studies reported that miR-223 regulates cancer cell invasion and migration through targeting ECT2 (34). Fabris et al. showed that miR-223 could inhibit the recurrence of breast cancer by mediating the EGF signaling pathway in their study (35). Citron et al. also showed that, in luminal breast cancer, the downregulation of miR-223 is crucial in the resistance of cancer cells to CDK4/6 inhibitors (36). These findings indicated that miR-223 may be critical in the progression of breast cancer. We validated that β-catenin is a direct target of miR-223 for the first time. We also observed that, in addition to protein function, CCT-3 mRNA also plays a critical role in breast cancer through miR-223 regulation. The downregulation of miR-223 in breast cancer is at least in part due to the overexpression of CCT-3. As Ala et al. described, the ceRNA network will be inoperative when the total number of mRNAs exceeds the number of their targeting miRNAs, resulting from the limited number of available miRNA molecules. Conversely, if the number of miRNA molecules exceeds the number of mRNA targets, the ceRNA network cross-regulation will not occur. Once the balance was disrupted, the miRNA–ceRNA crosstalk was affected, and diseases such as cancer may thus be promoted (37). We hypothesize that CCT-3 may be involved in a ceRNA network which includes other validated miR-223 target genes STMN-1, Caprin, and STAT5 (38–40). There are several algorithms to predict miRNA and target genes. Hence, there may exist several other potential miRNAs that bind to CCT-3 3′UTR, which are also valuable for research.

The article "Upregulation of CCT-3 Induces Breast Cancer Cell Proliferation Through miR-223 Competition and Wnt/β-Catenin Signaling Pathway Activation" was retracted in 2025. Reasons: original data or images not available; unreliable results or conclusions; concerns about the data; concerns about the images.

Wnt signaling is also associated with cancer cell migration and invasion. Therefore, the role of CCT-3/miR-223/β-catenin network in breast cancer cell proliferation, migration, and invasion can be explored in a further Wnt-related study.

In conclusion, our results suggest that CCT-3 is a potential oncogene with clinical significance. Understanding the role of CCT-3 in human breast cancer may provide new opportunities to develop novel therapeutic strategies such as chemical inhibitor, siRNA-based drugs, and Crispr/Cas9-based drugs. Furthermore, CCT-3 is also a potential diagnostic and prognostic biomarker for breast cancer.

## Data Availability Statement

The raw data supporting the conclusions of this article will be made available by the authors, without undue reservation.

## Ethics Statement

The animal study was reviewed and approved by ethics committee of the First People's Hospital of Chenzhou. The studies involving human participants were reviewed and approved by the ethics committee of the First People's Hospital of Chenzhou. The patients/participants provided their written informed consent to participate in this study.

## Author Contributions

HQ, FZ, and HD did the molecular and cellular experiments. XH and MH did the animal experiments. All the authors designed this research.

## Conflict of Interest

The authors declare that the research was conducted in the absence of any commercial or financial relationships that could be construed as a potential conflict of interest.

## Supplementary Material

Supplementary Figure 1 **(A)** RNA levels of CCT-3 in 1,106 breast cancer samples, including 998 cancer samples and 108 normal samples. Data from http://starbase.sysu.edu.cn/index.php. **(B)** Kaplan–Meier curves with univariate analyses (log-rank) for patients with breast cancer with low CCT-3-expressing tumors (*n* = 1,250) vs. high CCT-3-expressing tumors (*n* = 1,065). Data from http://kmplot.com/analysis/index.php?p=updates. The expression range of the probe is 57–17,685, and the database split patients by the median value of the probe. **(C)** RNA levels of miR-223 in 770 breast cancer samples, including 683 cancer samples and 87 normal samples. Data from http://starbase.sysu.edu.cn/index.php. **(D)** RNA level correlation between CCT-3 and miR-223 in 748 breast cancer samples. Data from http://starbase.sysu.edu.cn/index.php.

The article "Upregulation of CCT-3 Induces Breast Cancer Cell Proliferation Through miR-223 Competition and Wnt/β-Catenin Signaling Pathway Activation" was retracted in 2025. Reasons: original data or images not available; unreliable results or conclusions; concerns about the data; concerns about the images.

Supplementary Table 1 Clinicopathological characteristics of patient sample and expression of CCT3 in Breast Cancer.

Supplementary Table 2 Correlation between CCT3 expression and cliniclpathologic characteristics of Breast Cancer.
